# Clinical Nursing Paths Benefit Patient Outcomes Undergoing Transcatheter Arterial Chemoembolization for Hepatocellular Carcinoma

**DOI:** 10.1155/2022/4655293

**Published:** 2022-06-20

**Authors:** Jing Gu, Yao Liang

**Affiliations:** Zhangjiagang First People's Hospital, No. 68, Jiyang West Road, Zhangjiagang, Suzhou 215600, Jiangsu Province, China

## Abstract

**Objective:**

The purpose of the study is to investigate patient outcomes of transcatheter arterial chemoembolization (TACE) for hepatocellular carcinoma (HCC) under clinical nursing paths (CNP) and whether the application of CNP can be a protective factor against the recurrence of HCC.

**Methods:**

The study comprised of 48 patients who received TACE for HCC under the CNP (assigned into the CNP group) and 41 who received TACE for HCC under the routine care (assigned into the control group). Their treatment safety, pain, and psychology were compared. The nursing satisfaction and quality of life were investigated when patients were discharged from the hospital. A 6-month follow-up was performed to analyze the related factors affecting disease recurrence.

**Results:**

In the CNP group, the incidence rate of total adverse reactions, VAS scores, SAS and SDA scores were lower, but conversely, the satisfaction and SF-36 scores were higher than those in the control group (*P* < 0.05). Logistic regression analysis revealed that advanced TNM stage, larger tumor diameter, greater Child-Pugh classification, and the presence of peripheral blood vessel invasion were independent risk factors of HCC recurrence (*P* < 0.05).

**Conclusion:**

The study demonstrated that CNP intervention can improve the safety and quality of life of patients undergoing TACE for HCC and reduce their negative emotions and pain feelings, which is worthy of clinical application.

## 1. Introduction 

Hepatocellular carcinoma (HCC), as one of the common malignancies, has a high incidence and mortality worldwide [1]. The initial onset of HCC is hidden and most of the diseases have no obvious symptoms. When patients have symptoms such as pain in the liver area, the disease is mostly in the middle and late stage, which poses a serious threat to their life and health [2]. HCC is a malignancy in the liver, which is related to drinking, viral hepatitis, eating moldy food, and heredity [3]. It is possible to cure the disease in the early stage, the treatment in the middle and late stage is relatively complex, and the efficacy in the early stage of intersection is quite different [4]. At the moment, an interventional therapy is a nonsurgical method and the first choice for advanced HCC patients [5]. Embolic agents and anticancer drugs are injected into the hepatic artery through femoral artery intubation to achieve the efficacy. In clinical practice, the transcatheter arterial chemoembolization (TACE) has been widely accepted as the first option for nonsurgical HCC treatment [6]. However, patients with HCC often suffer from poor response to TACE therapy.

Previous data reflected that, during TACE, effective nursing intervention has a positive effect on improving the efficacy of TACE. It can not only help patients relieve the pain during treatment but can also decrease complications after invasive treatment [7]. Clinically, new nursing models are constantly being developed to meet the needs of nursing intervention in different diseases. The clinical nursing path (CNP) is a new nursing model, which is characterized by comprehensive clinical nursing experience, more targeted service to each patient, the development of its own nursing path, and more comprehensive and detailed help to patients [8]. It has been proved to exhibit excellent clinical values in treating many diseases, such as stroke [9, 10]. However, there is still much controversy about the nursing intervention after TACE for HCC. This research focuses on patient outcomes of TACE for HCC under CNP and whether the application of CNP can be a protective factor against the recurrence of HCC.

## 2. Materials and Method

### 2.1. Patient Data Collection

The study retrospectively analyzed 89 HCC patients who received TACE in our hospital from July 2020 to May 2021. Among them, 48 receiving TACE under CNP after admission were assigned into the CNP group and 41 receiving TACE under routine care were assigned into the control group. The review of patient data was approved by the Ethics Committee of our hospital, and all included patients signed informed consent forms. Included patients must be diagnosed with HCC by the pathology department of our hospital, meet requirements to receive TACE, and have expected survival ≥6 months. The Child-Pugh classification and TNM stage of HCC were confirmed according to the previous report [11]. The exclusion criteria were as follows: patients with other malignancies; patients with multiple chronic diseases; patients with other cardiovascular and cerebrovascular diseases; patients with organ dysfunction; patients with drug allergy; patients with mental illness or physical disability who are unable to take care of themselves; patients with surgical taboos; and patients transferred from one hospital to another.

### 2.2. The Protocols of CNP Intervention

After admission, all the patients were treated by the same surgical team in our hospital, and the control group was given routine care after operation. In brief, the nursing staff should explain the treatment methods before operation, remind patients of the precautions, help them make preoperative preparations, monitor their vital signs in time after operation, guide patients to take medication according to the doctor's orders, communicate with the attending doctor in time for the adverse symptoms after operation, and give intervention. Meanwhile, appropriate psychological counseling and health guidance were given to patients. The CNP group was given CNP intervention: A CNP team was established, the head nurse of the department served as the team leader, the head nurse of the ward and 2 nursing team leaders served as team members, and a chief physician of the vascular interventional department provided consultant support. By reviewing the references and related materials and synthesizing the opinions of the team members, we formulated a work implementation table, and the nursing content is implemented according to the schedule (Table 1). Furthermore, the staff should communicate with the attending physician in time when there is an abnormal situation, assist him to complete the treatment, and sign the completed work every day.

### 2.3. Follow-Up

Patients were followed up for a period of 6 months, and the follow-up was conducted in hospital referral with an interval of no more than 2 months. The cut-off event was the recurrence of the disease and the deadline was January 10, 2022. The prognosis and recurrence of the disease were recorded.

### 2.4. Pittsburgh Sleep Quality Index (PSQI)

The PSQI was employed to evaluate sleep quality in the past month [12], consisting of 19 questions belonging to seven component scores: subjective sleep quality, sleep latency, sleep duration, habitual sleep efficiency, sleep disturbances, use of sleeping medication, and daytime dysfunction. Each question has a range of 0 to 3 points and one global score has a range of 0 to 21 points, “0” indicating no difficulty and “21” indicating severe difficulties in all areas. A global score ≥5 indicates a high risk of reduced sleep quality.

### 2.5. Visual Analog Scale (VAS)

The pain of patients was assessed using the VAS scoring system which is a standard and verified 10-point scale for pain self-report [13]. The system score has a range of 0 to 10, with a score of 0 representing no pain and a score of 10 representing the highest pain level.

### 2.6. Self-Rating Anxiety Scale (SAS) and Self-Rating Depression Scale (SDS)

The SAS was used to assess the anxiety of patients and its validity and reliability have been demonstrated previously [14]. The SAS contains 20 components to reflect symptoms of anxiety, yielding a total score ranging from 20 to 80. A score of 50 is recommended as a score to identify students with anxiety.

The SDS was used to assess the depressive symptoms of patients [15], which covers 20 items to describe symptoms of depression, yielding a total score ranging from 4 to 80 points. Depression is classified as mild with a score between 53 and 62, moderate with a score between 63 and 72, or severe with a score of not less than 72.

### 2.7. Short Form Health Survey (SF-36) and Nursing Satisfaction

The quality of life of patients was assessed using the SF-36, which is a 36-item, which is a validated self-reported survey with component scores for the mental and the physical health domains [16], involving physical functioning, role-physical, bodily pain, general health, vitality, social functioning, role-emotional, and mental health. A higher SF-36 domain score indicates better quality of life.

An anonymous nursing satisfaction questionnaire was performed to investigate the nursing satisfaction of patients when they were discharged from hospital.

### 2.8. Statistical Analysis

The data were statistically analyzed by using SPSS (IBM Corp. Released 2016. IBM SPSS Statistics for Windows, Version 24.0. USA). The counting data of both groups were expressed as number (rate) and compared by using chi-square test; The measurement data were represented as mean ± standard deviation and compared by using *t*-test. The independent risk factors of HCC recurrence after TACE were assessed by logistic regression analysis. The significant differences were statistically marked as *P* < 0.05.

## 3. Results

### 3.1. CNP Intervention Prevents the Incidence of Adverse Reactions after TACE

We first collected demographic data of HCC patients in the CNP group and control group and statistically analyzed whether the two groups were comparable. There was no obvious difference in terms of age, BMI, and gender between both groups (*P* > 0.05), indicating that the two groups were comparable (Table 2). The incidence of adverse reactions such as gastrointestinal reaction, nausea and vomiting, liver pain, urinary retention, fever, and bleeding were recorded in the CNP group and control group after TACE. We found the total incidence of adverse reactions was 6.25% in the CNP group and 21.95% in the control group. The incidence of adverse reactions in the CNP group was lower than that in the control group, and the difference was statistically significant (*P* < 0.05). The CNP group had a shorter length of hospital stay with reduced hospitalization costs compared with the control group (Table 3).

### 3.2. CNP Intervention Improved Sleep Quality and Reduced Pain Feeling after TACE

The sleep quality and pain scores of HCC patients in the CNP group and control group after TACE were assessed by the PSQI and VAS score system. It was found that the sleep quality of patients in the CNP group was better but the pain scores was lower than that in the control group (*P* < 0.05) (Figure 1).

### 3.3. CNP Intervention Reduced Anxiety and Depression after TACE

The degree of anxiety and depression in both groups were tested through the SAS and SDS scores. It reflected that the SAS and SDS scores in the CNP group were lower than those in the control group (*P* < 0.05) (Figure 2).

### 3.4. CNP Intervention Increased Nursing Satisfaction and Improved Quality of Life after TACE

The nursing satisfaction of patients was collected. It denoted that those patients in the CNP group were more satisfied with the survey results than those in the control group (*P* < 0.05), but there was no marked difference in the number of satisfied, needing improvement, and dissatisfied cases (*P* > 0.05) (Table 4). The SF-36 quality of life scale was conducted to evaluate the quality of life of patients after treatment from eight items: physiological function, role-physical, bodily pain, general health, vitality, social function, role-emotional, and mental health. It was found that the scores of all items in the CNP group were higher than those in the control group (*P* < 0.05) (Table 5).

### 3.5. Univariate Analysis of Prognostic Factors of HCC Recurrence after TACE

As of January 10, 2022, we have successfully followed up 89 HCC patients. Among them, 16 had disease recurrence. A univariate analysis was carried out between recurrent and nonrecurrent patients. It displayed that BMI, gender, living environment, educational level, and nationality were not the single factors affecting HCC recurrence (*P* > 0.05), but age, TNM stage, the Child-Pugh grade of liver function, and invasion of peripheral vessels were those affecting HCC recurrence after TACE (*P* < 0.05) (Table 6).

### 3.6. Multivariate Analysis of Independent Prognostic Factors of HCC Recurrence after TACE

The age, TNM stage, the Child-Pugh grade of liver function, and invasion of peripheral vessels were assigned into multivariate analysis. The prognostic recurrence was taken as the dependent variable and the predictive index as the covariable for logistic regression analysis. The predictive model satisfied the Hosmer–Lemeshow test for goodness-of-fit (*P*=0.60) and was therefore well calibrated. It revealed that age was not independently tied to prognostic recurrence (*P* > 0.05), but TNM stage, the Child-Pugh grade of liver function, and invasion of peripheral blood vessels were independent prognostic factors of HCC recurrence after TACE (*P* < 0.05) (Table 7).

## 4. Discussion

As a high-incidence malignancy in clinical practice, HCC is characterized by a relatively insidious initial onset and patients are diagnosed in the middle and late stages. So, it is difficult to treat and has an unsatisfactory prognosis [17]. Currently, interventional therapy for HCC is the first choice for advanced HCC treatment, and the implementation of effective clinical nursing interventions in interventional therapy can stabilize the condition of patients, reduce the occurrence of treatment complications, and promote better postoperative recovery [18]. Liao et al. pointed out that CNP could improve the cognitive function and quality of life in hypertensive cerebral infarction patients [19] whereas Zhang et al. clarified that CNP had an improved significance for percutaneous coronary intervention [20]. All these have laid a reliable foundation for implementing CNP in TACE for HCC. CNP intervention is a kind of patient-centered targeted nursing service, which has achieved remarkable results in diseases such as children's kidney disease and hip replacement, which can effectively improve their recovery [21, 22]. However, the application effect of interventional therapy for HCC is rarely reported. Hence, this research has an important reference significance for future clinical treatment by exploring the application results of interventional therapy for HCC under CNP.

As we all know, infection after interventional therapy has always been a hot topic in clinical research, and it is also one of the key factors affecting the efficacy and prognosis of patients [23]. Thus, we first compared the adverse reactions during treatment between patients. It showed that the incidence of adverse reactions in the CNP group was lower than that in the control group, indicating that TACE for HCC under CNP has higher safety. In a previous study, we also found that CNP could reduce the incidence of adverse reactions after bronchoscopy [24], which can also corroborate the results of this experiment and further illustrate the excellent application value of CNP. In the process of implementing CNP intervention, it is necessary to establish a nursing path table with patients as the core. Then, based on the table, the nursing staff can effectively improve the work efficiency and strengthen the sense of responsibility. Besides, because nurses are given professional training in advance, their professionalism can be improved, so as to increase patients' trust in nurses and satisfaction in nursing [25]. This can also be verified when we evaluate their pain.

In addition, due to the lack of awareness of interventional therapy in the process of HCC treatment, it is easy to restrict the effect of interventional therapy and adversely affect the rehabilitation of patients [26]. In the CNP intervention, through the in-depth study of medicine and nursing, a clear treatment and nursing process is adopted to make patients have a sense of trust in health care. On the one hand, it increases the trust between doctors and patients and improves the relationship between nurses and patients, so as to improve patients' compliance with treatment and nursing. On the other, the decrease of SAS and SDS scores in the CNP group also shows that CNP intervention is more helpful to the negative psychology of patients. We believe that this is because the CNP intervention is a nursing model for HCC diagnosis and treatment. It has a standardized nursing process, and nursing intervention is carried out in accordance with the nursing process in the hospital and after discharge, so that the knowledge education before treatment enables patients and their families to fully understand the process of interventional therapy and the purpose of treatment, so as to reduce their anxiety. Psychological burden increases patients' confidence in treatment and their satisfaction with treatment. Nursing interventions such as diet, hospital environment, daily nursing, and exercise not only enable patients to recover faster but also improve their awareness of disease and rehabilitation treatment, which is vital for prognosis and life. Quality is also valuable. In the quality-of-life assessment of patients after treatment, we also observed that the scores of those in the CNP group were increased, which verified our idea. Moreover, Han and Yu also found that CNP intervention could improve the quality of life of stroke patients [27], which is consistent with the results of this experiment. Finally, in the prognostic follow up, we found that the TNM stage, Child-Pugh grade of liver function, and invasion of peripheral blood vessels were all risk factors for disease recurrence after TACE for HCC, which was also consistent with the results of previous studies [28, 29]. This also suggests that we need to pay attention to the abovementioned conditions of patients when implementing TACE for HCC, so as to reduce the probability of recurrence and improve their prognosis.

Nevertheless, due to the lack of authoritative clinical guidelines for nursing intervention in TACE for HCC, it is not ruled out that there may be other nursing methods that are also suitable for TACE for HCC and can also achieve excellent results. In this study, only conventional nursing is used as a control, and we need to include a comparative study with the nursing model in the follow up to obtain more representative results. In addition, the cycle of this research is short, and the number of cases included and the follow-up cycle need to be improved in order to evaluate the long-term prognosis of CNP intervention after TACE for HCC.

In summary, CNP intervention can improve the safety and quality of life of patients with TACE for HCC and reduce their negative emotion and pain feeling, which is worthy of clinical application. The TNM stage, Child-Pugh grade of liver function, and invasion of peripheral blood vessels are the risk factors of disease recurrence after TACE for HCC.

## Figures and Tables

**Figure 1:** PSQI scores reflecting sleep quality (a) and VAS scores reflecting pain feelings (b) of the CNP group and control group after TACE. ^*∗*^ indicates *P* < 0.05.

**Figure 2:** SAS scores reflecting the anxiety and SDS scores reflecting the depression of the CNP group and control group after TACE. ^*∗*^ indicates *P* < 0.05.

**Table 1:** The protocols of CNP intervention.

Time	Nursing strategy
On the first day of admission	(a) Education before therapy: introduction to environment, system, personnel, disease information, and treatment.
	(b) Routine examination of admission: blood routine and physical sign examination.
	(c) Dietary guidance: low fat, low sugar, high protein, high vitamins, no smoking and alcohol.
	(d) Create medical records.

On the second day of hospitalization	(a) Routine biochemical examination: liver and kidney function and blood coagulation function.
	(b) B-ultrasonic examination of liver, gallbladder, pancreas, and spleen.
	(c) Introduce the matters needing attention before and after interventional therapy.
	(d) Sign surgery consent.

On the day of treatment	(a) Enter the intervention room for treatment accompanied by medical staff.
	(b) Postoperative dietary guidance: avoid greasy foods within 2 h after surgery.
	(c) Observe whether there is bleeding, exudate, and hematoma at the intervention site, use sandbags for acute compression to stop bleeding, and monitor the pulse of the dorsal artery of the foot.
	(d) Ankle pump exercise was performed after 24 h and 6 h of limb immobilization after operation.
	(e) Closely monitor the changes of vital signs.
	(f) Use painkillers according to the condition of patients.

On the first day after treatment	(a) The recovery of the involved limb was observed and the bandage was removed in 24 h.
	(b) Guide correct rehabilitation activities and assist patients to complete simple activities such as getting out of bed.
	(c) Observe postoperative complications.
	(d) Regular examination of the liver and kidney function.

On the second and third day after treatment	(a) Continue the infusion as directed by the doctor.
	(b) Evaluate the spirit and state of mind of patients.
	(c) Strengthen patients' ability of freedom movement and self-care.
	(d) Pay attention to vital signs and complications.

On the day of discharge	(a) Blood routine and coagulation function test.
	(b) Issue contact cards, introduce the time of revisit after discharge, emphasize the guidelines and matters needing attention in drug use, and establish follow-up.

**Table 2:** Demographic data of HCC patients in the CNP group and control group.

	CNP group (*n* = 48)	Control group (*n* = 41)	*t* or *χ*^2^	*P*
Age	52.4 ± 3.5	52.2 ± 2.9	0.291	0.772
BMI (kg/cm^2^)	26.16 ± 3.39	25.67 ± 2.68	0.747	0.457

Gender			0.443	0.506
Male	32 (66.67%)	30 (73.17%)		
Female	16 (33.33%)	11 (26.83%)		

Living environment			0.064	0.800
Urban	28 (58.33%)	25 (60.98%)		
Rural	20 (41.67%)	16 (39.02%)		

Educational level			0.041	0.839
<High school	33 (68.75%)	29 (70.73%)		
≥High school	15 (31.25%)	12 (29.27%)		

Nationality			0.414	0.520
Han	46 (95.83%)	38 (92.68%)		
Minority	2 (4.17%)	3 (7.32%)		

TNM staging			0.027	0.870
I-II	32 (66.67%)	28 (68.29%)		
III-IV	16 (33.33%)	13 (31.71%)		

Child-Pugh classification			1.080	0.583
Class A	32 (66.67%)	23 (56.10%)		
Class B	12 (25.00%)	13 (31.71%)		
Class C	4 (8.33%)	5 (12.20%)		

Invasion of peripheral blood vessels			0.182	0.670
No	37 (77.08%)	30 (73.17%)		
Yes	11 (22.92%)	11 (26.83%)		

**Table 3:** The incidence of adverse reactions, length of hospital stay, and hospitalization costs between both groups.

	CNP group (*n* = 48)	Control group (*n* = 41)	*t* or *χ*^2^	*P*
Gastrointestinal reaction	1 (2.08%)	2 (4.88%)		
Nausea and vomiting	1 (2.08%)	1 (2.44%)		
Liver pain	0 (0.00%)	2 (4.88%)		
Urinary retention	0 (0.00%)	1 (2.44%)		
Fever	1 (2.08%)	2 (4.88%)		
Bleeding	0 (0.00%)	1 (2.44%)		
Total incidence	3 (6.25%)	9 (21.95%)	4.673	0.031
Length of hospital stay	10.03 ± 1.51	12.32 ± 2.68	5.04	<0.001
Hospitalization costs	4989.33 ± 116.20	6209.52 ± 163.78	40.77	<0.001

**Table 4:** Nursing satisfaction of the CNP group and control group after TACE.

	CNP group (*n* = 48)	Control group (*n* = 41)	*χ* ^2^	*P*
Very satisfied	27 (56.25%)	11 (26.83%)	7.823	0.005
Satisfied	17 (35.42%)	20 (48.78%)	1.626	0.202
Needing improvement	3 (6.25%)	6 (14.63%)	1.710	0.191
Dissatisfied	1 (2.08%)	4 (9.76%)	2.455	0.117

**Table 5:** Two groups of SF-36 quality of life scale.

	CNP group (*n* = 48)	Control group (*n* = 41)	*t*	*P*
Physiological function	70.96 ± 9.99	64.34 ± 8.85	3.283	0.002
Role-physical	67.00 ± 7.44	62.29 ± 9.15	2.678	0.009
Bodily pain	68.67 ± 7.44	64.61 ± 8.27	2.437	0.017
General health	71.04 ± 7.54	63.05 ± 8.54	4.688	<0.001
Vitality	74.85 ± 9.11	66.98 ± 9.89	3.905	<0.001
Social function	73.15 ± 6.51	65.02 ± 6.57	5.848	<0.001
Role-emotional	83.63 ± 8.02	73.61 ± 12.62	4.534	<0.001
Mental health	80.06 ± 7.49	73.37 ± 8.06	4.055	<0.001

**Table 6:** Univariate analysis of prognostic recurrence in patients.

	Recurrence (*n* = 16)	Nonrecurrence (*n* = 73)	*t* or *χ*^2^	*P*
Age	54.9 ± 2.8	51.8 ± 3.1	3.682	<0.001
BMI (kg/cm^2^)	26.33 ± 1.99	25.85 ± 3.27	0.563	0.575

Gender			0.474	0.491
Male	10 (62.50%)	52 (71.23%)		
Female	6 (37.50%)	21 (28.77%)		

Living environment			0.088	0.767
Urban	9 (56.25%)	44 (60.27%)		
Rural	7 (43.75%)	29 (39.73%)		

Educational level			0.263	0.608
<High school	12 (75.00%)	50 (68.49%)		
≥High school	4 (25.00%)	23 (31.51%)		

Nationality			1.161	0.281
Han	0 (0.00%)	5 (6.85%)		
Minority	16 (100.0%)	68 (93.15%)		

TNM staging			15.980	<0.001
I-II	4 (25.00%)	56 (76.71%)		
III-IV	12 (75.00%)	17 (23.29%)		

Child-Pugh classification			22.020	<0.001
Class A	3 (18.75%)	52 (71.23%)		
Class B	7 (43.75%)	18 (24.66%)		
Class C	6 (37.50%)	3 (4.11%)		

Invasion of peripheral blood vessels			22.060	<0.001
No	5 (31.25%)	63 (86.30%)		
Yes	11 (68.75%)	10 (13.70%)		

Way of nursing			2.120	0.145
Normal nursing	10 (62.50%)	31 (42.47%)		
CNP nursing	6 (37.50%)	42 (57.53%)		

**Table 7:** Multivariate analysis of factors affecting patients' prognosis and recurrence.

	Β	S.E.	Wald *χ*^2^	HR	95% CI	*P*
Age	−1.042	1.054	0.994	0.342	0.040–2.841	0.241
TNM staging	−2.142	0.842	15.931	1.113	0.421–1.624	<0.001
Child-Pugh classification	2.142	1.340	22.413	5.541	0.771–10.426	<0.001
Invasion of peripheral blood vessels	2.142	1.521	14.242	2.241	1.410–6.814	<0.001

## Data Availability

The data used to support the findings of this study are included within the article.
